# Primary Investigation of Deep Learning Models for Japanese “Group Classification” of Whole-Slide Images of Gastric Endoscopic Biopsy

**DOI:** 10.1155/2022/6899448

**Published:** 2022-09-26

**Authors:** Xiaoya Fan, Lihui Yu, Xin Qi, Xue Lin, Junjun Zhao, Dong Wang, Jing Zhang

**Affiliations:** ^1^School of Software, Key Laboratory for Ubiquitous Network and Service Software of Liaoning Province, Dalian University of Technology, Dalian, Liaoning, China; ^2^Dalian Municipal Central Hospital, Dalian, Liaoning, China

## Abstract

**Background:**

Accurate pathological diagnosis of gastric endoscopic biopsy could greatly improve the opportunity of early diagnosis and treatment of gastric cancer. The Japanese “Group classification” of gastric biopsy corresponds well with the endoscopic diagnostic system and can guide clinical treatment. However, severe shortage of pathologists and their heavy workload limit the diagnostic accuracy. This study presents the first attempt to investigate the applicability and effectiveness of AI-aided system for automated Japanese “Group classification” of gastric endoscopic biopsy.

**Methods:**

In total, 260 whole-slide images of gastric endoscopic biopsy were collected from Dalian Municipal Central Hospital from January 2015 to January 2021. These images were annotated by experienced pathologists according to the Japanese “Group classification.” Five popular convolutional neural networks, i.e., VGG16, VGG19, ResNet50, Xception, and InceptionV3 were trained and tested. The performance of the models was compared in terms of widely used metrics, namely, AUC (area under the receiver operating characteristic curve, i.e., ROC curve), accuracy, recall, precision, and F1 score.

**Results:**

Results showed that ResNet50 achieved the best performance with accuracy 93.16% and AUC 0.994.

**Conclusion:**

Our results demonstrated the applicability and effectiveness of DL-based system for automated Japanese “Group classification” of gastric endoscopic biopsy.

## 1. Background

Gastric cancer has long been acknowledged as a severe public health problem across the globe [1] with a 5-year survival rate of lower than 40% [2]. Despite the decrease of mortality over the past few decades in some countries, it remains the fourth leading cause of cancer death worldwide [3] and third in China [4]. In China, it is still highly prevalent and accounts for over 40% of new cases in the world [3, 4]. Most gastric cancer cases are diagnosed at an advanced stage due to its atypical symptoms in early stage and late aggressive behaviors [5]. The situation is more severe in China, where more than 60% of patients were diagnosed at an advanced stage [6]. However, the treatment options are often limited at this stage, resulting in unsatisfactory prognosis [7]. Early diagnosis of gastric cancer enables early clinical intervention, thus improving prognosis and survival rate. Currently, timely and correct diagnosis of gastric cancer relies heavily on pathological examination of gastric biopsy tissue, which is performed by highly trained pathologists with an optical microscopy. However, this process is tedious and time-consuming. Moreover, the accuracy of pathological diagnosis of gastric biopsy is quite limited [4] due to the shortage of pathologists worldwide. Such shortage leads to heavy workload for pathologists and possible errors in diagnosis.

Therefore, there is a great need for automated and accurate pathology diagnosis of gastric cancer. Several applications of deep learning (DL) models have emerged in digital pathology image analysis. The common task is either binary classification task as tumor detection or three-way classification task as cancer classification. For instance, Wang et al. [8] proposed GastricNet, a DL-based framework for automatic gastric cancer identification. The model achieved 100% accuracy for slice-based classification, outperforming the state-of-the-art networks like DenseNet and ResNet. Leon et al. [9] proposed two independent approaches based on convolutional neural network (CNN) for gastric cancer detection using histopathological image samples. The first one analyzed the morphological features of the whole image. The second one analyzed the local characteristic properties. The histopathological image was classified as either benign or malignant. Qu et al. [10] performed the same task with a transfer learning strategy. The model was first pretrained with ImageNet and further fine-tuned with a well-annotated benign/malignant dataset. A detection accuracy of up to 89.72% was achieved, showing the promise of automated gastric cancer detection. On the other hand, Sharma et al. [11] explored the deep learning methods for classification in H&E-stained histopathological whole slide images (WSIs) of gastric carcinoma. The WSIs were classified as HER2+ tumor, HER2- tumor, or nontumor. The model achieved an overall accuracy of 0.6690. More recently, Iizuka et al. [12] investigated the feasibility of CNNs and recurrent neural networks (RNNs) for classifying WSI into adenocarcinoma, adenoma, and nonneoplastic, achieving area under the curves (AUCs) up to 0.97 and 0.99 for gastric adenocarcinoma and adenoma, respectively. The work described above suggests that DL models are promising for pathological image analysis for gastric cancer. However, clinical application remains challenging. The ultimate purpose of automated pathological image analysis is to better serve for decision making in treatment. However, this work does not immediately translate to clinic decisions.

In China, the majority of pathologists are trained with *WHO classification* [13] while most treatment options are adopted from Japan [4, 5] with reference to the *Japanese Gastric Cancer Treatment Guidelines* [14] (Japanese guidelines). However, the pathological classification adopted in Japanese guidelines is the “group classification” of gastric biopsy specimens (Groups 1~5), rather than WHO classification. Thereby, the pathologists and gastroenterologists speak different languages, and the pathological diagnosis does not correspond well with clinical treatment decisions.

In this paper, the feasibility of deep learning models for automated Japanese “Group classification” of WSIs of gastric endoscopic biopsy was investigated. Five popular DL models, VGG-16 [15], VGG-19 [15], ResNet-50 [16], Xception [17], and InceptionV3 [18], were trained and compared. Results showed that ResNet50 achieved the best performance with an accuracy of 93.16% and an AUC of 0.994. To the best of our knowledge, this is the first attempt to investigate the applicability and effectiveness of AI-aided system for pathological group classification of human gastric epithelial lesions.

## 2. Methods

### 2.1. Whole-Slide Image Preparation

In total, 260 cases of gastric endoscopic biopsy from 173 patients (128 males and 45 females, aged from 27 to 92 years old, mean ± std: 65.2 ± 11.4) with human gastric epithelial lesions were collected from Dalian Municipal Central Hospital from January 2015 to January 2021. The WSIs were stained with hematoxylin and eosin (H&E) and further produced at ×40 magnification (0.238 *μ*m/pixel) by the digital scanner (KF-PRO-005). All procedures performed in studies involving human participants were approved by the Medical Ethics Committee of Dalian Municipal Central Hospital and in accordance with the 1964 Helsinki declaration and its later amendments or comparable ethical standards. Informed written consent was also obtained from individual participants included in the study. The workflow of the study is illustrated in Figure 1.

### 2.2. Annotation Procedure

All the WSIs were annotated by two experienced pathologists using an open-source annotation tool *labelme* (https://github.com/wkentaro/labelme). According to the Japanese “Group classification,” gastric endoscopic biopsy can be classified as 5 groups (see Figure 2 for illustration). The description of the 5 groups is shown in Table 1. Briefly, it defines Group 1 as normal tissue or nonneoplastic lesion tissue, Group 2 as tissue that is difficult to make diagnosis between neoplastic and nonneoplastic lesions, Group 3 as adenoma, Group 4 as tissue with neoplastic lesion that is suspected to be carcinoma, and Group 5 as tissue with carcinoma [14].

The annotation tool, *labelme*, enables the pathologists to segment a WSI into various regions and label each region with the group they belong to. It has to be noted that different regions from a single WSI could be labeled as different groups, whereas a single region can only be labeled as a single group. The annotation process was accomplished by two pathologists. Pathologist 1 first drew the outline of each region and annotated with Groups 1~5. The initial annotation was then modified, confirmed, or verified by a senior pathologist. An example of WSI with final annotation is illustrated in Figure 3. The region outlined in red was annotated as Group 5, while the region outlined in green was annotated as Group 1. The remaining regions that were not outlined were the regions that are hard to classify.

### 2.3. Preprocessing and Datasets

A big challenge faced in computational pathology is the huge size of a WSI. A single image can contain hundreds of millions of pixels. To apply deep learning models, a WSI image was first segmented into small tiles with 400 × 400 pixel size. The tiles with a tissue area less than 50% were discarded. In clinical practice, in order to increase diagnostic accuracy, pathologists often observe the specimens under various magnifications of the view (40×, 100×, 200×, and 400×). Therefore, we varied the size of the tiles from 400 × 400 pixel, 600 × 600 pixel, 800 × 800 pixel to 1000 × 1000 pixel and established 5 datasets consisting of tiles with different sizes (see Table 2). All datasets underwent the tile selection process described above.

### 2.4. Model Training, Testing, and Evaluation

Each dataset was split into a training set (60%), validation set (20%), and testing set (20%). To avoid data imbalance, the splitting process was done within each group. Five popular models were trained, i.e., VGG16, VGG19, ResNet50, Xception, and InceptionV3. Standard data augmentation techniques (such as reflection, rotation, and shift) and early stopping were employed to avoid overfitting. TensorFlow was used as the framework to build DL models. All models were trained/tested on one Nvidia GeForce RTX 2080Ti 8 GB GPU.

Commonly used metrics, namely, overall accuracy (Acc) and area under the receiver operator characteristic (ROC) curve (AUC), were used to evaluate the performance of the models, which were calculated from comparing model prediction with the annotation of pathologists. The accuracy, recall, precision, and F1 score were also calculated for each group to provide detailed information of model performance.

Acc represents the overall accuracy, which was defined as the percentage of correctly predicted tiles in all tiles.

The recall for Group *i* was defined as

(1) $$\begin{array}{c} \text{Recall}=\frac{\text{TP}}{\text{TP}+\text{FN}}, \end{array}$$

where TP (true positive) is the number of tiles that were annotated as Group *i* by pathologists and correctly predicted as Group *i* by the model; FN (false negative) is the number of tiles that were annotated as Group *i* but predicted incorrectly as any other groups by the model. It represents the percentage of tiles that were correctly predicted by the model in all tiles annotated as Group *i* by pathologists.

The precision for Group *i* was defined as

(2) $$\begin{array}{c} \text{Precision}=\frac{\text{TP}}{\text{TP}+\text{FP}}, \end{array}$$

where FP (false positive) is the number of tiles that were predicted as Group *i* but annotated as any other groups by pathologists. It stands for the percentage of tiles that were annotated as Group *i* by pathologists in all tiles that were predicted as Group *i* by the model.

The F1 score, a metric that combines both precision and recall, was defined as

(3) $$\begin{array}{c} \text{F}1\text{ score}=\frac{2\times \text{precision}\times \text{recall}}{\text{Precision}+\text{recall}}. \end{array}$$

## 3. Results

### 3.1. Among the Five Model Architectures, ResNet50 Performs the Best

We first compared the performance of five different models trained with Dataset 1 (see Table 3). Among the five models, ResNet50 achieved the best performance with an AUC of 0.988 and an Acc of 89.5%, followed by VGG16 and VGG19 with an AUC of 0.970 and 0.949, respectively. We further analyzed the accuracy, recall, precision, and F1 score of the five models for each group individually (see Figure 4). Results showed that ResNet50 achieved 90.33%, 81.56%, 88.33%, 81.15%, and 95.18% recall for Groups 1~5, respectively, leading all the other models for all groups. As also can be seen, ResNet50 outperformed all other models in terms of all metrics (higher green bars in Figure 4), except precision for Group 1, which is slightly lower compared to VGG16 (89.08% compared to 90.22%).

### 3.2. The Best Performance Was Achieved with Dataset 5 with Mixed Size of Tiles

We further tested the performance of the ResNet50 models trained with different datasets. The AUC and Acc are listed in Table 4. As can be seen, ResNet50 performed the best when trained with Dataset 5 with an AUC of 0.994 and an Acc of 93.16%, which consists of tiles with mixed sizes. Apart from the overall AUC and Acc, we also calculated the accuracy, recall, precision, and F1 score of ResNet50 models for each group trained with different datasets (Figure 5). Results showed that ResNet50 achieved the highest accuracy, recall, precision, and F1 score for all groups when trained on Dataset 5 (higher green bars in Figure 5), except the highest recall for Group 5, which was achieved when the model was trained on Dataset 3.  Figure 6 shows the normalized confusion matrix of ResNet50 trained on Dataset 5 to better illustrate the model performance.

## 4. Discussion

The present study is the first attempt to investigate the feasibility of deep learning models for automated Japanese “Group classification” based on WSIs. Specifically, we trained 5 popular CNN models, namely, VGG16, VGG19, ResNet50, Xception, and InceptionV3. Results showed that ResNet50 achieved the leading performance in terms of AUC and Acc. This is not surprising since comprehensive empirical evidence has shown that residual network can gain accuracy from considerably increased depth. To apply DL models to huge WSIs, each WSI was first segmented into small tiles. We varied the size of tiles and built five datasets that constitute tiles of different sizes (see Table 2). In clinic, pathologists observe the biopsy under various magnifications of view to enhance diagnosis. Similarly, a dataset with mixed sized tiles was also constructed in this work. We further trained ResNet50 with different datasets. Results showed that when trained with mixed sized tiles (Dataset 5), the model achieved the best performance, with an AUC of 0.994 and an Acc of 93.16%. With tiles of different sizes, the model is able to “see” the samples at various spatial scales, as the pathologists observe the biopsy under various magnifications of view. Our results suggest that DL models for automated Group classification of neoplastic lesion biopsy is promising and could help relief the workload of pathologists and increase diagnosis accuracy.

A closer investigation suggested that such improvement lies in a much higher recall for Group 2 (88.48% compared to 81.56%, 74.68%, 64.63%, and 67.51%) and Group 4 (90.70% compared to 81.15%, 83.21%, 76.27%, and 79.64%) and a fairly higher recall for Group 3 (91.07% compared to 88.33%, 87.61%, 85.14%, and 81.32%). The correct recognition of Groups 2~4 gastric biopsy is challenging in clinical practice. Meanwhile, it is critical for early detection of gastric cancer, enabling good prognosis with proper intervention. Therefore, higher recall for Groups 2~4 is of high clinical importance. Our results suggest that training the model with mixed sized tiles enables a higher recall for Groups 2~4.

In addition, our results suggest that the size of tiles has an effect on the model performance. An interesting trend revealed by our results is that the model degenerates when trained with bigger tiles. Two possible reasons may explain this. First, when segmented into big-sized tiles, the number of tiles is smaller. The samples in the training set could be insufficient for model training, leading to underfitting of the model. Second, the big-sized tiles are more likely to contain unwanted information, increasing the difficulty of model training.

There is currently no standardized treatment protocol that is globally accepted, and clinical practice alters across countries. This is mainly due to the fact that gastric cancer populations from different countries have distinct etiology, epidemiological characteristics, and clinicopathological features, especially between the East and the West [2, 4, 5]. There are several pathological diagnosis systems of gastric cancer around the world. Two main systems are the “WHO classification of tumors of digestive system” [13] and the Japanese “Group classification” [14]. Most pathologists in China are trained with the “WHO classification” while the gastroenterologists are trained with the Japanese guidelines. Such discrepancy causes a reduction in collaboration efficiency between the pathologists and gastroenterologists. Therefore, current pathological diagnosis system in China does not fully play its due role in guiding clinical treatment. The Japanese “Group classification,” on the other hand, corresponds well with the endoscopic diagnostic system and could provide direct guidance for clinical treatment. Another problem that cannot be ignored in China is that the pathologists are extremely in short. Therefore, AI-aided automatic system for Japanese “Group classification” of gastric epithelial lesions is of clinical importance and the present study is the first attempt. If validated, such a system could be applied, not only to relieve the workforce of pathologists and improve their diagnosis accuracy but also to better translate pathological diagnosis to clinical practice.

To the best of our knowledge, the present study is the first to investigate the feasibility of automated Japanese “Group classification” of gastric biopsies based on pathological images. Automated pathological image analysis for human gastric epithelial lesions is not a novel topic. Most studies focus on early cancer diagnosis or cancer classification and treat the task as a binary [9, 10] or three-way classification problem [19]. For instance, Qu et al. [10] proposed a step-wise fine-tuning approach for gastric pathology image classification, where the model was first pretrained with ImageNet and further fine-tuned with a well-annotated benign/malignant dataset. Similarly, Leon et al. [9] proposed a CNN-based approach to classify gastric histopathological images as benign or malignant. On the other hand, Li et al. [19] proposed a DL-based approach for early diagnosis of gastric cancer, where non-precancerous lesion, precancerous lesion, and gastric cancer were automatedly differentiated. Sharma et al. [11] proposed a convolutional neural network for cancer classification based on immunohistochemical response and achieved 0.669 accuracy, in which the WSIs of surgical sections were classified as HER2+ tumor, HER2- tumor, or nontumor.

A common limitation of DL models for medical applications is that their interpretability is very weak. Their decision should be suggestive or assisted, rather than deterministic. However, they are still quite helpful. One important application of the present study is to quickly screen out Group 1 and Group 5 biopsy, which is defined as normal tissue or nonneoplastic lesion tissue and carcinoma, respectively. Although the pathological diagnosis of Group 1 and Group 5 is relatively easy, it still takes time. Such automated screening could greatly reduce the workload of pathologists so that they have more time spending on other suspicious specimens, thus increasing the diagnosis accuracy, as well as efficiency. ResNet50 achieved 7.24% false-negative rate for Group 1 and 4.32% false-positive rate for Group 5, respectively, suggesting its potential to be applied as so. The false-positive rate and false-negative rate for each group are provided in Table 5. The false-negative rate for Group 5 indicates the rate of missed diagnosis of carcinoma, which can have a more negative effect on the patient. Therefore, a low value is highly expected. Our results showed 3.18% false-negative rate for Group 5, which is acceptable for an assistive screening system. Moreover, the inference time for one WSI is about 30 seconds, which is shorter than conventional diagnosis by pathologists with a microscope. The elapsed training time is about 7 hours.

One limitation of the present study is that all WSIs were collected from one center and produced by an identical digital scanner. WSIs from multiple centers with various digital scanners should be included for further validation of this approach.

## 5. Conclusions

This paper presents the first attempt to investigate the applicability of convolutional neural networks for automated Japanese “Group classification” of WSIs of gastric endoscopic biopsy. Five popular CNNs were trained and tested. Results showed that ResNet50 achieved the best performance with an accuracy of 93.16% and an AUC of 0.994. Our results demonstrated the applicability and effectiveness of DL-based system for automated Japanese “Group classification” of gastric endoscopic biopsy.

## Figures and Tables

**Figure 1:** Workflow of the study.

**Figure 2:** Typical examples of Groups 1~5 according to the Japanese “Group classification.” Framed in the left corner of each subfigure is the typical appearance of the corresponding class.

**Figure 3:** An example of annotated WSI, segmented with *labelme*. Outlined in red was annotated as Group 5 while in green was annotated as Group 1.

**Figure 4:** Performance (accuracy, recall, precision, and F1 score) of five different models for each group evaluated on the test set. All models were trained on Dataset 1. The values of the metrics for ResNet50 are highlighted above the corresponding green bars.

**Figure 5:** Performance (accuracy, recall, precision, and F1 score) of ResNet50 evaluated on the test set. The models were trained on five different datasets. The values of the metrics for ResNet50 trained on Dataset 5 are highlighted above the green bars.

**Figure 6:** Normalized confusion matrix of ResNet50 on the test set. The model was trained on Dataset 5.

**Table 1:** Description of Japanese “Group classification”.

Group	Description
Group 1	Normal tissue or nonneoplastic lesion tissue
Group 2	Difficult to make diagnosis between neoplastic and nonneoplastic lesions
Group 3	Adenoma
Group 4	Can be diagnosed as neoplastic lesion and is suspected to be carcinoma
Group 5	Carcinoma

**Table 2:** Information of datasets.

	Group 1	Group 2	Group 3	Group 4	Group 5
Number of WSIs	166	84	45	68	58
Dataset 1 (400 × 400)	45001	10274	17999	20845	41521
Dataset 2 (600 × 600)	21430	4307	7584	8967	17834
Dataset 3 (800 × 800)	10875	2291	4204	4931	9944
Dataset 4 (1000 × 1000)	7243	1387	2652	3044	6318
Dataset 5 (mixed size^∗^)	39548	7985	14440	16942	34096

^∗^Tiles with various sizes (600 × 600, 800 × 800, and 1000 × 1000) were mixed to construct Dataset 5.

**Table 3:** Test accuracy of five different models^∗^.

Model	AUC	Acc (%)
ResNet50	0.988	89.5
VGG16	0.970	83.1
VGG19	0.949	76.6
Xception	0.894	66.2
InceptionV3	0.881	63.0

∗The models were trained on Dataset 1.

**Table 4:** AUC and accuracy of ResNet-50 models trained on different datasets.

Dataset	AUC	Acc (%)
Dataset 1 (400 × 400)	0.988	89.48%
Dataset 2 (600 × 600)	0.989	90.64%
Dataset 3 (800 × 800)	0.983	88.09%
Dataset 4 (1000 × 1000)	0.979	87.21%
Dataset 5 (mixed size)	0.994	93.16%

**Table 5:** The false-positive rate (FPR) and false-negative rate (FNR) of each group.

	Group 1	Group 2	Group 3	Group 4	Group 5
FPR	5.94%	16.93%	5.60%	10.01%	4.32%
FNR	7.24%	11.52%	8.93%	9.30%	3.18%

## Data Availability

The datasets used and/or analyzed during the current study are available from the corresponding authors on reasonable request.

## Abbreviations

AI: Artificial intelligence
AUC: Area under the ROC curve
CNN: Convolutional neural network
DL: Deep learning
FN: False negative
FP: False positive
HER2+: Human epidermal growth factor receptor-2 positive
HER2-: Human epidermal growth factor receptor-2 negative
H&E: Hematoxylin and eosin
RNN: Recurrent neural network
ROC: Receiver operating characteristic curve
WHO: World Health Organization
WSI: Whole slide image
TP: True positive.
